# Knowledge of and Compliance with Surviving Sepsis Campaign Guidelines among Anesthesiologists: A Nationwide Survey in China

This article has been retracted.

**DOI:** 10.1155/2021/1877166

**Published:** 2021-09-22

**Authors:** Hui Li, Xiangyang Yu, Rui Zhou, Ya Wang, Xuedi Zhang, Shengwen Song, Qinghua Chen, Baoli Cheng, Xiangming Fang

**Affiliations:** Department of Anesthesiology, The First Affiliated Hospital, School of Medicine, Zhejiang University, Hangzhou, China

## Abstract

We aimed to describe anesthesiologists' knowledge of and compliance with the Surviving Sepsis Campaign (SSC) guidelines in the perioperative management of patients with sepsis in China. We designed a questionnaire-based, cross-sectional survey. We sent out online questionnaires during 2019 to evaluate whether anesthesiologists in China were familiar with and applied SSC guidelines in perioperative management. We also compared anesthesiologists' knowledge of and compliance with the guidelines among different levels of hospital. In this study, we obtained 971 responses from anesthesiology departments across China. The survey responses showed that 39.0% of anesthesiologists rated their knowledge of the SSC guidelines as being “very familiar” or at least “somewhat familiar.” In total, 68.9% of respondents chose “Initial fluid resuscitation followed by frequent hemodynamic reassessment” as their therapy strategy for patients with septic shock; 62.0% of anesthesiologists chose lactate as a marker of initial resuscitation in clinical practice, and 39.1% thought bundle therapy needed to be started within 1 hour of sepsis diagnosis. A total of 37.1% and 27.1% of respondents chose hydroxyethyl starches and gelatins, respectively, as the preferred fluids for septic shock. As the first choice of vasopressors in patients with sepsis, 727 (74.9%) anesthesiologists chose the correct answer (norepinephrine). Anesthesiologists from tertiary hospitals (class A) had greater familiarity and compliance with the SSC guidelines than those from other hospitals (*P* < 0.001). In summary, anesthesiologists in China have some knowledge of the SSC guidelines and tend to practice in keeping with these guidelines. However, for some items, anesthesiologists are not up to date with the latest version of the SSC guidelines. The popularity of these guidelines is not homogenous among different levels of hospital. Anesthesiologists must strengthen their knowledge of the SSC guidelines and update their practice in a regular and timely manner, especially in other tertiary and primary hospitals.

## 1. Introduction

As one of the most challenging medical problems, sepsis is defined as life-threatening organ dysfunction induced by an uncontrolled host response to infection [1, 2]. It is estimated that there are 31.5 million new patients with sepsis and 5.3 million deaths every year worldwide, making sepsis a serious public health burden [3]. The Surviving Sepsis Campaign (SSC), a multinational collaboration led by the Society for Critical Care Medicine, was launched in 2002 and is devoted to improving the outcomes of sepsis and septic shock [2, 4]. In the SSC, four editions of clinical guidelines were formulated on the basis of existing clinical evidence, in 2004, 2008, 2012, and 2016, aiming to guide clinicians in diagnosing and treating patients with sepsis. Increasing evidence has indicated that implementation of the SSC guidelines is associated with improved outcomes in both adults and children with sepsis [5–8].

Sepsis is an important cause of death in critically ill surgical patients. A study in the United States showed that the incidence of sepsis in patients undergoing surgery is 20.2% [9]. Our team also conducted a multicenter, nationwide, epidemiological survey of surgical patients with sepsis in China, the results of which showed that the overall hospital mortality rate owing to sepsis with organ dysfunction was as high as 48.7% [10]. Anesthesiologists play an important role in the perioperative management of surgical patients with sepsis. The 2018 SSC bundle combined the previous 3-h and 6-h bundles into a single “1-hour bundle,” which highlights early diagnosis and early treatment to a greater degree [11]. This change places more stringent requirements on anesthesiologists who treat patients with sepsis undergoing emergency surgery because these are most likely to be in the time window of the“1-hour bundle.” However, compliance with the SSC guidelines in the initial management of surgical patients with sepsis among anesthesiologists has not been described. For years, many scientists have been committed to researching and constantly striving to publicize and popularize the positive role of the SSC guidelines in perioperative patients with sepsis. However, whether the mastery and application of the SSC guidelines by anesthesiologists is improving remains a question of great concern.

In the current study, we administered questionnaires during 2019 to investigate knowledge and compliance with the SSC guidelines among anesthesiologists across China. We also compared anesthesiologists' knowledge and compliance with the guidelines among different levels of hospital.

## 2. Materials and Methods

### 2.1. Study Design

This study was designed as a questionnaire-based, cross-sectional survey. The questionnaire was designed and pretested using the Tencent questionnaire website (https://wj.qq.com/mine.html). The questionnaire was linked via the website and WeChat and then disseminated to anesthesiologists in all provinces of China. We designed an 18-item questionnaire, based on the 2016 guidelines and 2018 updates. We mainly focused on fluid administration and the use of vasoactive drugs for patients with sepsis. The questionnaires comprised three main aspects: (1) demographic information, including age, regional distribution, degree and title, years of working as an anesthesiologist, and hospital level; (2) anesthesiologists' overall familiarity with the SSC guidelines and how well they had mastered the guidelines; and (3) anesthesiologists' compliance with and application of the guidelines in their clinical practice.

### 2.2. Participants and Procedure

The questionnaires were submitted from 31 July to 25 August 2019. Respondents were anesthesiologists from across China who were willing to participate in the survey. No incentives to complete the survey were offered. The respondents were free to withdraw at any time. Any questionnaires with incomplete answers were excluded from the statistical analysis. The questionnaires were completed anonymously and voluntarily in the survey.

### 2.3. Statistical Analysis

Data analysis was performed using IBM SPSS 20.0 for Windows (IBM Corp., Armonk, NY, USA). Categorical variables are presented as percentages, and the differences among levels of hospital were analyzed using the *χ*^2^ test combined with the Bonferroni test. Group comparisons for ranked data among different levels of hospital were analyzed using Kruskal–Wallis one-way analysis of variance (k samples). We considered a difference to be statistically significant with *P* < 0.05.

## 3. Results

### 3.1. Basic Characteristics

Data from 971 anesthesiologists were analyzed.  Table 1 shows the basic characteristics of anesthesiologists, including hospital level, number of operations per year for patients with sepsis, and anesthesiologists' degrees, title, and years working as an anesthesiologist. To explore the differences among levels of hospital, we divided hospitals where anesthesiologists worked into four groups: university-affiliated tertiary hospitals (class A), nonaffiliated tertiary hospitals (class A), other tertiary hospitals (class B and C), and primary hospitals. There were 462 (47.6%), 193 (19.9%), 111 (11.4%), and 205 (21.1%) survey respondents from university-affiliated tertiary hospitals, nonaffiliated tertiary hospitals, other tertiary hospitals, and primary hospitals, respectively.

### 3.2. Anesthesiologists' Overall Familiarity and Compliance with the Latest SSC Guidelines

A total of 379 (39.0%) anesthesiologists rated their knowledge of the Surviving Sepsis Guidelines as being “very familiar” or at least “somewhat familiar” (Table 2). In total, 524 (54.0%) anesthesiologists always or usually administered fluid therapy according to SSC guidelines, and 349 (35.9%) sometimes administered fluid therapy according to SSC guidelines (Table 2). As for the percentage of survey respondents who used the guidelines correctly in fluid therapy, 669 (68.9%) thought that additional fluids should be guided by reassessment of hemodynamic status following initial fluid resuscitation (updated in the 2016 guidelines and 2018 SSC bundle); however, 198 (20.4%) had outdated knowledge and chose early goal-directed therapy (Table 2). Among respondents, 871 (89.7%) thought that fluid selection during general elective surgery differed from fluid resuscitation in septic shock (Table 2). Most anesthesiologists felt that the 2018 guidelines were suitable for perioperative fluid therapy, with 675 (69.6%) rating the suitability as 4–5 on a scale ranging from 1 (not suitable) to 5 (very suitable) (Table 2).

### 3.3. Anesthesiologists' Knowledge and Practice regarding 2016 SSC Guidelines and 2018 Updates

To understand how well Chinese anesthesiologists have mastered the SSC guidelines, we asked a series of questions on the survey based on the 2016 guidelines and 2018 SSC bundles. When asked about the content of bundle therapy after the update to the guidelines in 2018, the correct responses—measure lactate level, begin fluid resuscitation immediately and stress fluid reactivity assessment, obtain blood cultures, administer vasopressors if necessary, and administer broad-spectrum antibiotics—were correctly chosen by 77.2%, 84.4%, 73.9%, 81.9%, and 66.1% of respondents, respectively (Table 3). A total of 529 (54.5%) and 680 (70%) respondents to the survey chose mean arterial pressure (MAP) and lactate level as markers of initial resuscitation, respectively (Table 3). For the correct target value of initial resuscitation markers, 41.2% of anesthesiologists considered lactate concentration of ≤2 mmol/L as the target value for effective fluid resuscitation, and 286 (29.5%) selected MAP of ≥65 mmHg as the target value for effective fluid resuscitation (Table 3). The 2018 SSC stresses that bundle therapy needs to be started within 1 hour after the diagnosis of sepsis, and 380 (39.1%) of survey respondents chose the correct answer (Table 3). Regarding the first choice of vasopressors for patients with sepsis, 727 (74.9%) of anesthesiologists chose the correct answer (norepinephrine) (Table 3).

To further clarify practical application of the SSC guidelines among anesthesiologists in China, we investigated their responses regarding fluid choice and markers of initial resuscitation. As shown in Table 4, 85.6% of survey respondents chose Ringer's lactate solution, 65.8% chose hydroxyethyl starches, and 41.1% chose polygeline as the three preferred fluids in elective surgery for patients without sepsis. Acetate Ringer's solution (52.9%), lactate Ringer's solution (50.6%), and hydroxyethyl starches (37.1%) were selected as the three preferred fluids for resuscitation in patients with sepsis (Table 4). The anesthesiologists indicated that the three most important factors affecting fluid selection were the availability of fluids, protocol of the department or hospital, and the SSC guidelines (Table 4). Respondents chose urine output (692 [71.3%]), MAP (605 [62.3%]), and lactate level (602 [62.0%]) as the three preferred target markers of initial resuscitation (Table 4). Anesthesiologists indicated that the three most important factors affecting their choice were difficulty with indicator detection, restrictions on routine testing in the department or hospital, and the SSC guidelines (Table 4).

### 3.4. Comparison of Anesthesiologists' Knowledge of and Compliance with the SSC Guidelines among Different Levels of Hospital

The results showed that anesthesiologists from tertiary hospitals (class A) (including university-affiliated hospitals and nonaffiliated hospitals) had greater familiarity and compliance with the SSC guidelines in comparison with those from other tertiary and primary hospitals (*P* < 0.001; Table 5; Figures 1(a) and 1(b)). As for whether fluid selection for patients with sepsis differed from fluid selection in elective surgery and whether the 2018 guidelines were considered suitable for perioperative fluid therapy, no difference was found among the four hospital-level groups (*P* > 0.05; Table 5; Figure 1(c)). Anesthesiologists from tertiary hospitals (class A) had a higher percentage of correct answers for the first choice of vasopressors compared with those from other hospitals (*P* < 0.001; Table 5; Figure 1(d)). Anesthesiologists from university-affiliated tertiary hospitals had a higher percentage of correct answers for the target value of MAP than those from other tertiary and primary hospitals (*P* < 0.05; Table 5; Figure 1(e)), but comparisons among other groups showed no significant differences (*P* > 0.05; Table 5; Figure 1(e)). Similarly, anesthesiologists from university-affiliated tertiary hospitals had a higher percentage of correct answers for the target value of lactate than those from primary hospitals (*P* < 0.05; Table 5; Figure 1(f)), but comparisons among other groups did not show any significant differences (*P* > 0.05; Table 5; Figure 1(f)).

## 4. Discussion

This study was designed to investigate the knowledge of and compliance with the SSC guidelines among anesthesiologists and to analyze differences among hospital levels. Sepsis is a serious threat to human health and a global medical problem. There are more than 750,000 patients diagnosed with sepsis in the United States each year, and its mortality is as high as 28.6% [12]. Similarly, an epidemiological survey in China showed that the in-hospital mortality rate of sepsis is 20.6%, and the standardized mortality rate is 79/100,000 [13]. These data reveal high morbidity and mortality of sepsis, which has drawn extensive attention in the medical field. Because of the pathophysiological particularity of sepsis, patients usually have circulatory instability, lung injury, and other organ dysfunction, which makes perioperative anesthesia management complex and challenging [14]. The SSC guidelines provide an important reference for the management of patients with sepsis. Several studies have observed adherence to the SSC guidelines by physicians in emergency medicine (EM), critical care medicine (CCM), and internal medicine (IM) [15, 16]. However, compliance with the SSC guidelines by anesthesiologists in the initial management of surgical patients with sepsis has not been investigated.

In this study, we described anesthesiologists' knowledge of and compliance with SSC guidelines in China. The results showed that 39.0% of anesthesiologists rated their knowledge of the SSC guidelines as being “very familiar” or at least “somewhat familiar,” and 68.9% thought that additional fluids should be guided by reassessment of hemodynamic status following initial fluid resuscitation (updates in the 2016 guidelines and 2018 SSC bundle). For the first choice of vasopressors in patients with sepsis, 727 (74.9%) of respondents chose the correct answer (norepinephrine). A survey [15] among EM, IM, and CCM physicians in the United States evaluated whether they were familiar with and incorporating the SSC guidelines into their practice. The results showed that significant differences existed among the three specialties. CCM physicians followed more elements of the SSC guidelines than IM and EM physicians, such as measuring serum lactate and preferring norepinephrine as the first vasopressor. Another survey conducted in Scotland also indicated differences for early fluid and vasopressor management of sepsis between Scottish ICM and EM consultants [16].

In recent years, the role of plasma lactic acid level detection has received greater attention. Several randomized controlled trials have evaluated lactate-guided resuscitation in patients with sepsis, and the results have suggested a significant reduction in mortality [17–20]. Svetolik's team found that 79.7%, 66.0%, and 60.3% of EM, IM, and CCM physicians, respectively, always or usually used serum lactate as a marker of initial resuscitation [15]. In our study, 70% of anesthesiologists used lactate levels as the marker of initial resuscitation, and 62.0% chose lactate as a marker of initial resuscitation in clinical practice. These data are similar to those of Svetolik's report.

Recent SSC guidelines recommend crystalloid solutions for fluid resuscitation in patients with sepsis or septic shock and albumin in patients requiring substantial amounts of crystalloids [2]. Use of hydroxyethyl starches results in a higher risk of renal replacement therapy and death [2, 21]. However, 37.1% and 27.1% of survey respondents in the current study chose hydroxyethyl starches and gelatins, respectively, as their preferred colloidal fluid for septic shock. These data revealed that the knowledge and practice of Chinese anesthesiologists are not up to date with the latest version of the SSC guidelines. Chinese anesthesiologists are required to urgently improve their knowledge of the SSC guidelines and update their clinical practice.

When we compared respondents' knowledge of and compliance with the guidelines among different levels of hospital, we found that anesthesiologists from tertiary hospitals (Class A) had greater familiarity and compliance with the SSC guidelines than those from other hospitals. These data proved that popularity of the guidelines is not homogenous among different levels of hospital. The possible reason is that anesthesiologists in tertiary hospitals (Class A) have more opportunities to treat critically ill patients with sepsis, which motivates them to be up to date with the latest guidelines. Moreover, the medical facilities in tertiary hospitals (Class A) are more complete and advanced, which ensures that anesthesiologists conduct clinical practice in accordance with the guidelines. Therefore, a positive attitude toward learning and practice, as well as abundant medical resources, considerably affects anesthesiologists' knowledge and practice.

Several recommendations are suggested to improve the knowledge of and compliance with SSC guidelines among Chinese anesthesiologists. First, publicize and popularize the role of SSC guidelines in perioperative administration through the national academic annual meetings, lectures of further education in colleges, and daily morning courses in the Department of Anesthesiology. Second, develop mobile phone APP for providing a pathway to consult relevant content of the updated SSC guidelines. Third, efforts should be made to disseminate relevant material to different levels of hospitals for sustained dissemination and implementation of updated guidelines.

There are two limitations in the present study. First, we were unable to administer the questionnaire in remote areas owing to the unavailability of multimedia equipment; however, these areas account for a very small proportion of China. Second, the anesthesiologists received the website links to the questionnaires and voluntarily completed the questionnaires; therefore, the recruitment of survey respondents may be biased toward anesthesiologists who are more interested in the SSC guidelines.

## 5. Conclusion

Our survey study revealed that anesthesiologists in China have some knowledge of the SSC guidelines and tend to practice in keeping with the SSC guidelines. However, for some items of the guidelines, anesthesiologists are not up to date with the latest SSC guidelines in terms of their knowledge and practice. Popularity of the guidelines is not homogenous among different levels of hospital. Anesthesiologists are required to strengthen their knowledge of the SSC guidelines and update their practice in a regular and timely manner.

## Figures and Tables

**Figure 1:** Comparison of anesthesiologists' knowledge and compliance with SSC guidelines among different levels of hospitals. ^*∗*^*P* < 0.05 vs. university-affiliated hospital group. ^#^*P* < 0.05 vs. nonaffiliated hospital group. (a) Familiarity with SSC guidelines. (b) Compliance with SSC guidelines. (c) Fluids selection. (d) What's the target value of MAP？. (e) What's the target value of lactate level. (f) What's the first choice of vasopressors.

**Table 1:** The basic characteristics of participants and their hospitals in 2019.

Characteristic	2019 (*n* = 971)
Hospital levels	
University-affiliated hospital	462 (47.6%)
Nonaffiliated hospital	193 (19.9%)
Other tertiary hospitals	111 (11.4%)
Primary hospital	205 (21.1%)
Number of operations per year for patients with septic patients	
<50	497 (51.2%)
50–150	278 (28.6%)
150–300	98 (10.1%)
>300	98 (10.1%)
Degree	
Doctor	123 (12.7%)
Master	330 (34.0%)
Bachelor	461 (47.5%)
Junior college	57 (5.9%)
Title	
Senior	158 (16.3%))
Deputy senior	277 (28.5%)
Intermediate	343 (35.3%)
Junior	193 (19.9%)
Years of working as anesthesiologists	
＜3 years	93 (9.6%)
3–5 years	85 (8.8%)
5–10 years	174 (17.9%)
＞10 years	619 (63.8%)

All data were presented as absolute values and percentages of total number of responses from anesthesia department.

**Table 2:** Anesthesiologists' overall familiarity and compliance with the latest SSC guidelines in China.

Assessment items	*n* (%)
Familiarity with SSC guidelines	
Very familiar	72 (7.4%)
Somewhat familiar	307 (31.6%)
General knowledge	485 (50.0%)
Don't know	107 (11.0%)
Compliance with SSC guidelines	
Always	138 (14.2%)
Usually	386 (39.8%)
Sometimes	349 (35.9%)
Never	98 (10.1%)
Therapy strategy for septic shock	
EGDT	198 (20.4%)
Initial fluid resuscitation followed by frequent hemodynamic reassessment	669 (68.9%)
Empiric therapy	104 (10.7%)
Whether fluids selection for sepsis shock is different from selective operation or not	
Yes	871 (89.7%)
No	100 (10.3%)
Whether 2018 guidelines are suitable for the perioperative fluid therapy ranging from 1 (not suitable) to 5 (very suitable)	
1	7 (0.7%)
2	39 (4.0%)
3	250 (25.8%)
4	392 (40.4%)
5	283 (29.2%)

All data were presented as absolute values and percentages of total number of responses from the Department of Anesthesiology. EGDT, early goal-directed therapy.

**Table 3:** Anesthesiologist's knowledge of the 2016 SSC guidelines and 2018 update in China.

Assessment items	*n* (%)
What elements are included in bundle therapy after the update of SSC guidelines in 2018?	
Measure lactate level	750 (77.2%)
Obtain blood cultures	718 (73.9%)
Begin fluid resuscitation immediately and stress fluid reactivity assessment	819 (84.4%)
Apply vasopressors if necessary	795 (81.9%)
Administer broad-spectrum antibiotics	642 (66.1%)
What are the markers of initial resuscitation in the 2018 SSC guidelines?	
MAP	529 (54.5%)
CVP	439 (45.2%)
Lactate levels	680 (70%)
Urine output	588 (60.6%)
SvO_2_ or ScvO_2_	675 (69.5%)
How many hours bundle therapy needs to be started once sepsis is diagnosed?	
Percentage of correct answer (1 hour)	380 (39.1%)
What's the target value of MAP?	
Percentage of correct answer (≥65 mmHg)	286 (29.5%)
What's the target value of lactate level?	
Percentage of correct answer (≤2 mmol/L)	400 (41.2%)
What's the first choice of vasopressors?	
Percentage of correct answer (norepinephrine)	727 (74.9%)

All data were presented as absolute values and percentages of total number of responses from the Department of Anesthesiology. MAP, mean arterial pressure; CVP, central venous pressure; SvO_2_, mixed venous oxygen saturation; ScvO_2_, superior vena cava oxygenation saturation.

**Table 4:** Anesthesiologist's practice of the 2016 SSC guidelines and 2018 update in China.

Assessment items	*n* (%)
The preferred markers of initial resuscitation	
MAP	605 (62.3%)
CVP	462 (47.6%)
Lactate levels	602 (62.0%)
Urine output	692 (71.3%)
SvO_2_ or ScvO_2_	324 (33.4%)
The preferred fluids in selective operation	
Lactic Ringer's solution	831 (85.6%)
Acetic Ringer's solution	317 (32.7%)
Physiological saline	347 (35.7%)
Hydroxyethyl starches	639 (65.8%)
Polygeline	399 (41.1%)
Concentrated erythrocyte	116 (12.0%)
The preferred fluids for septic shock	
Lactic Ringer's solution	491 (50.6%)
Acetic Ringer's solution	514 (52.9%)
Physiological saline	305 (31.4%)
Hydroxyethyl starches	360 (37.1%)
Polygeline	263 (27.1%)
Albumin	398 (41%)
Plasma	314 (32.3%)
Concentrated erythrocyte	131 (13.5%)
The most important factors affecting their fluid selection	
Economic aspects	295 (30.4%)
Availability of fluids	798 (82.2%)
Habits of the department or hospital	675 (69.5%)
Guidelines	740 (76.2%)
Surgeons' decisions	106 (10.9%)
The most important factors affecting their choice of markers of initial resuscitation?	
Difficulty of detection	626 (64.5%)
Instructions from superior doctor	238 (24.5%)
Restrictions on routine testing items in the department or hospital	724 (74.6%)
Guidelines	647 (66.6%)
Personal experience	483 (49.7%)

All data were presented as absolute values and percentages of total number of responses from the Department of Anesthesiology. Options with a selection rate less than 10% are not presented in the table. MAP, mean arterial pressure; CVP, central venous pressure; SvO_2_, mixed venous oxygen saturation; ScvO_2_, superior vena cava oxygenation saturation.

**Table 5:** Comparison of anesthesiologists' knowledge and compliance with SSC guidelines among different levels of hospitals.

Assessment items	Tertiary hospital (class a)		Other tertiary hospitals	Primary hospital	*P*
	University-affiliated hospital	Nonaffiliated hospital			
Familiarity with SSC guidelines					<0.001^*∗*^
Very familiar	49 (10.6%)	18 (9.3%)	0^*∗*#^	5 (2.4%)^*∗*#^	
Somewhat familiar	171 (37.0%)	62 (32.1%)	29 (26.1%)	45 (22.0%)	
General knowledge	206 (44.6%)	94 (48.7%)	67 (60.4%)	118 (57.6%)	
Don't know	36 (17.6%)	19 (9.8%)	15 (13.5%)	37 (18.0%)	
Compliance with SSC guidelines					<0.001^*∗*^
Always	76 (16.5%)	35 (18.1%)	8 (7.2%)^*∗*#^	19 (9.3%)^*∗*#^	
Usually	207 (44.8%)	83 (43.0%)	41 (36.9%)	55 (26.8%)	
Sometimes	148 (32.0%)	61 (31.6%)	49 (44.1%)	91 (44.4%)	
Never	31 (6.7%)	14 (7.3%)	13 (11.7%)	40 (19.5%)	
Whether fluids selection for sepsis shock is different from selective operation or not					= 0.673
Yes	410 (88.7%)	176 (91.2%)	102 (91.9%)	183 (89.3%)	
No	52 (11.3%)	17 (8.8%)	9 (8.1%)	22 (10.7%)	
What's the target value of MAP?					= 0.032^*∗*^
Percentage of correct answer (≥65 mmHg)	149 (32.3%)	58 (30.1%)	20 (18.0%)^*∗*^	59 (28.8%)	
What's the target value of lactate level?					= 0.014^*∗*^
Percentage of correct answer (≤2 mmol/L)	208 (45.0%)	85 (44.0%)	39 (35.1%)	68 (33.2%)^*∗*^	
What's the first choice of vasopressors?					<0.001^*∗*^
Percentage of correct answer (norepinephrine)	374 (81.0%)	161 (83.4%)	64 (57.7%)^*∗*#^	128 (62.4%)^*∗*#^	

^*∗*^ Significant difference among different levels of hospitals in 2019. Comparisons of familiarity and compliance were analyzed by Kruskal–Wallis one-way ANOVA (k samples), while other comparisons were analyzed by the *χ*^2^ test combined with the Bonferroni test. ^*∗*^*P* < 0.05 vs. university-affiliated hospital group. ^#^*P* < 0.05 vs. nonaffiliated hospital group. All data were presented as absolute values and percentages of total number of responses from the corresponding hospitals.

## Data Availability

All data generated or analyzed during this study are included in the article.

## Abbreviations

CVP: Central venous pressure
EGDT: Early goal-directed therapy
MAP: Mean arterial pressure
RCTs: Randomized controlled trials
ScvO_2_: Superior vena cava oxygenation saturation
SSC: The surviving sepsis campaign
SvO_2_: Mixed venous oxygen saturation.
